This article has been retracted.

# Basketball Data Analysis Using Spark Framework and *K*-Means Algorithm

**DOI:** 10.1155/2021/6393560

**Published:** 2021-07-27

**Authors:** Xijun Hong

**Affiliations:** College of Sports Science, Dali University, Dali 671003, Yunnan, China

## Abstract

With the rapid development, different information relating to sports may now be recorded forms of useful big data through wearable and sensing technology. Big data technology has become a pressing challenge to tackle in the present basketball training, which improves the effect of baseball analysis. In this study, we propose the Spark framework based on in-memory computing for big data processing. First, we use a new swarm intelligence optimization cuckoo search algorithm because the algorithm has fewer parameters, powerful global search ability, and support of fast convergence. Second, we apply the traditional *K*-clustering algorithm to improve the final output using clustering means in Spark distributed environment. Last, we examine the aspects that could lead to high-pressure game circumstances to study professional athletes' defensive performance. Both recruiters and trainers may use our technique to better understand essential player's qualities and eventually, to assess and improve a team's performance. The experimental findings reveal that the suggested approach outperforms previous methods in terms of clustering performance and practical utility. It has the greatest influence on the shooting training impact when moving, yielding complimentary outcomes in the training effect.

## 1. Introduction

Basketball is a sport that takes into account both individual skills and team collaboration [1–3]. The individual level of skill and team tactics are important in the game [4, 5]. Basketball's fundamental moves are dribbling, shooting, and triple laying. Dribbling among them is the most fundamental action in basketball, and shooting is the talent to score [6–9]. The correctness of fundamental motions influences the game's score. The outcome of shooting scores from professional basketball players is connected to angle and shooting strength, so that players' skills may develop with the practice of shooting motions [10–15]. There are certain faults in the player's training that do not comply with regular motions and the sensational analysis of their shootout. The long-term training of nonstandard motions will have a certain influence not only on the shooting outcomes but also on the players themselves. Basketball players' training is nowadays mostly targeted at fundamental motions. The typical training approach is that the coach speaks directly with the players and assesses how the movements are standardized by looking at the players' fire movements and the coach experience. Because this approach is based on the coach's intuitive feelings, there is no appropriate assessment and no criteria for the judgment of the players [16–18].

In recent years, with the rapid development of computer technology [19–21] and the popularity of the network, the data scale of sports especially basketball has increased sharply, and the data have grown exponentially. The rapid increase of data has promoted the advent of the era of sports big data. Faced with the increasing amount of data, emerging big data computing frameworks, represented by Hadoop [22] and Spark [23], have attracted more and more attention. Hadoop is an application platform for storing computing data. It consists of HDFS, YARN [24], MapReduce [25], and other components. It is an open-source project of the Apache Software Foundation. With the emergence of Hadoop, many enterprises, institutions, and governments have their own big data processing platforms. However, there are many shortcomings in the Hadoop framework. First, MapReduce will involve a large number of I/O operations in the process of iterative computation, which will lead to the waste of resources and seriously affect the performance of data processing. However, MapReduce operates independently in each iteration and has to wait for the result of the previous iteration, which needs to be stored in HDFS to judge whether the termination condition of iteration is met [26–28]. This wastes a lot of system performance. Finally, if the MapReduce framework needs to perform multiple functions, then multiple MapReduce programs need to be written, seriously degrading the performance of the MapReduce framework.

Due to its distributed features, cluster Spark has the great operational capability. It is very appropriate for mass data processing, along with Spark platform data mining techniques for the parallelization of classic data mining algorithms. The clustering analytical platform can successfully satisfy the data mining need for vast amounts of data in the background of data processing. Cluster analysis [29, 30] splits major data into many groups as one of the key study fields for data mining [31]. To make the data more comparable in the same cluster, assess the fixed characteristics between the various clusters [32]. The classical *K*-means clustering algorithm can be well applied in a distributed computing environment. When processing the data, the center of each class cluster, which requires several iterative computations, has to be continually calculated. Spark is an iterative computing memory-based framework, and it provides distinct benefits over MapReduce. The major contributions of the study are as follows to improve the *K*-means algorithm.

- The proposed scalable distributed Spark framework and *K*-means algorithm to analyze basketball data
- The proposed model considered the cuckoo search algorithm as a swarm intelligence algorithm to improve the traditional *K*-means clustering algorithm
- The proposed model implicitly distributes data, which has better global search ability and improves the clustering efficiency of the algorithm and the accuracy of the algorithm
- The proposed model considered nonlinearity in the dataset that is not easy to fall into local optimal using multistack processing layers and a nonlinear activation function for a better robustness model
- The performance of the suggested model is thoroughly assessed using the powerful computing abilities of the Spark cluster to handle the problem of basketball data mining more effectively in the context of enormous data

The rest of the study is organized as follows. In Section 2, a proposed system model design of the Apache Spark system is outlined. The evaluation method process analysis is conducted in Section 3. The experimental results and discussion is further summarized in Section 4. Finally, Section 5 concludes the study with a summary and future research directions.

## 2. Design of the Proposed Model

This section introduces the suggested model's design. The suggested model's design includes several components that are explained in depth.

### 2.1. Apache Spark Architecture

The overall architecture of Spark in a distributed environment is shown in Figure 1, which mainly includes two modules: driver and worker. The driver creates SparkContext by running the main () method in the application, creates the RDD, and performs the corresponding transformation actions on the RDD. SparkContext serves as a bridge between the data processing logic and the Spark cluster and is responsible for communicating with ClusterManager. ClusterManager makes unified scheduling of the cluster's resources. ClusterManager is allocated corresponding cluster computing resources for this task at the same time of launching executor to improve the efficiency of task scheduling as much as possible. The work of computing tasks in the cluster is taken care of by the WorkNode. When a computing task is executed on a cluster, the WorkNode starts an executor for the task. Then, the executor starts a thread pool that manages the task, where the task acts as the unit of computation on the executor. The driver will receive information from the executor about the health of the task, and finally, the executor will stop when all tasks have been executed. In addition, after years of accumulation, Spark has a series of components that constitute its ecosystem. The Spark core composition is shown in Figure 2.

The SparkCore is the cornerstone and core of the entire Spark ecosystem which mainly includes the creation of SparkContext, storage system, basic model architecture, task running process, and calculation engine. Spark SQL completes the processing function of structured data, and Spark Streaming can complete the function of real-time calculation, providing users with functions such as real-time data collection, real-time data calculation, and real-time data query. GraphX is a distributed graph computing processing tool provided by the Spark platform, which can be deployed in a distributed cluster. The framework has a rich graph computing mining API. Finally, MLib is a Spark machine learning component that makes machine learning easier and easier to implement, and it also facilitates the processing of larger-scale basketball sports data.

### 2.2. *K*-Means Algorithm

This section describes the basic flow of the *K*-means algorithm. First, determine the initial cluster center. Enter the number of cluster centers *k*, the dataset contains *n* cluster objects, select *k* data objects arbitrarily from the dataset *X*, and set it as the initial centroid *c*_1_, *c*_2_, *c*_3_,…, *c*_*k*_. Second, calculate the distance from the point *x*_*i*_(*i*=1,2,3,…, *n*) in the dataset to the *k* initial centroids. If ‖*x*_*i*_ − *c*_*j*_‖ < ‖*x*_*i*_ − *c*_*m*_‖, *j*=1,2,3,…, *k*,  *m*=1,2,3,…, *k* is satisfied, then *x*_*i*_ ∈ *C*_*j*_. Then, recalculate the centroid *c*_1_, *c*_2_, *c*_3_,…, *c*_*k*_ of the clusters again, and the calculation equation is as follows:

(1) $$\begin{array}{c} c_{i}=\frac{1}{n_{i}}\sum_{x_{j}\in C_{j}}^{x_{k}}x_{j}. \end{array}$$

Finally, if the distance between the new and prior centers of mass is zero, the new center of mass is equal to the old center of mass. If the difference between the two distances is less than the set threshold value, the calculation and algorithm are both halted; otherwise, the iterative computation is resumed by proceeding to Step 2.  Figure 3 depicts the flowchart of the original *K*-means clustering method.

### 2.3. Data Cluster Analysis

It has been used in a variety of disciplines. More and more individuals are learning about it and putting it to use. With the rapid expansion of the field of cluster analysis and the depth of research, numerous relevant publications concentrating on the study of clustering algorithms have been published. With the advent of the big data age, the effectiveness of classical clustering algorithms in processing data has been severely hampered due to the rising data scale. However, the introduction of distributed computing frameworks has resulted in very excellent practicality for analyzing and processing large amounts of data. Cluster analysis techniques are being used to import large data processing frameworks such as Hadoop, Spark, and others, and analysis and research are growing year after year. Although the big data framework offers users a high-level programming model, the model is implemented using the MapReduce computing model, and the MapReduce computing framework's abstract methods are only of two types: Map and Reduce. Without the use of distributed memory abstraction, data reuse which is the intermediate data between different computing wrote a stable file system (HDFS), for example, would generate data backup replication, disc I/O, and data serialization. It is extremely inefficient to operate if intermediate results from several computations must be reused. Spark transforms the data into RDD, a fault-tolerant and parallel data structure that enables users to explicitly store intermediate result datasets in memory and optimize data storage processing by regulating dataset division. RDD also has a robust API for modifying datasets. A wide range of operators meet the general analysis of the operation. Spark's usage of memory decreases the number of disc reads and writes during a calculation, making it significantly more computationally efficient than MapReduce, which is largely reliant on I/O. The current research trend is to apply the classic clustering method using the Spark distributed computing framework and alleviate the inadequacies of conventional clustering analysis by using the processing power of the cluster environment.

## 3. Evaluation Method

In this part, we show how to measure the performance of the suggested model. The confusion metrics are amongst the most extensively utilized techniques for identifying performance results by numerous academics. Stepping with both feet and then casting the basketball with a hand on your shoulder is the main point of the shot. The cognitive method adds a hop off the ground in comparison to the single-handed shot without taking it off. The jump's main movement holds the ball with both hands and places the hands-on on one side of the ball without shooting. The hands of the shooter on the back of the ball are knees bent, the hands hold the ball from the chest into the eyes, and the feet bounce up. Turn the elbow and roll the wrist down when you jump. When jumping to the highest point, stretch your forearm forward, throw your ball forth, and down with your wrist.

Correlation coefficient and mean absolute error are employed as assessment metrics in this work. The following formula is used to get the correlation coefficient.

(2) $$\begin{array}{c} \text{Corr}=\frac{1}{n}\sum_{i=1}^{n}\left(\frac{R_{i}-\bar{R}}{\sigma_{R}}\times \frac{P_{i}-\bar{P}}{\sigma_{P}}\right), \end{array}$$

where *n* is the actual mean and forecast mean for the psychotherapy level test sample correspondingly; The mean and standard deviation of the mean, as well as the standard deviation from *P* and standard deviation from, are represented by *R*. We have used the following equation to obtain the average absolute inaccuracy.

(3) $$\begin{array}{c} \text{MAE}=\frac{1}{n}\sum_{i=1}^{n}\left|R_{i}-P_{i}\right|. \end{array}$$

This is one of the most typical attack maneuvers in the basketball game, involving jumper, jumper, dribbling, and other operations. Many people often consider that, after repeated training, basketball players need the basic player to summarise their support experiences when they watch the jump basketball game for athletes to build the proper environment. There might be mistakes or myths in the athletes jumping on technical training. This is what we need to examine from the large basketball data.

## 4. Experiments and Results

### 4.1. Experimental Environment

We built up a Spark cluster, utilizing 5 physical processing nodes with default settings. The essential hardware and software requirements employed throughout the tests are explained in Table 1. All processing nodes have been set using the Ubuntu 18 LTS operating system, Spark 2.3.4 and Hadoop 2.7.3. The remaining three nodes were set up as the working nodes as the master node.

### 4.2. Scalability Analysis

To verify the clustering efficiency of the *K*-means clustering algorithm on basketball sports data, this study conducts a comparative experiment on scalability. The investigation of the scalability of the suggested model is shown in Figure 4 for both a multitude of dataset and a different number of processing nodes. Figures demonstrate that, with an increasing number of processing nodes, the proposed model time is considerably decreased.

In addition, we perform the original *K*-means classification method and the original *K*-means method in parallel. We run 20 tests each, and an algorithmic efficiency test of different algorithms was achieved.  Table 2 provides the shortest runtime for 20 experiments with datasets of different sizes, the longest runtime and the average run time of the algorithm. According to the data in Table 2, the serial *K*-means algorithm has the minimum clustering execution time of 12.36 seconds in the DATA1 dataset, while the parallel *K*-means algorithm has the longest execution time. Therefore, the serial *K*-means algorithm is superior to the parallel *K*-means algorithm. In DATA2 and DATA3, the parallel *K*-means algorithm is superior to the serial *K*-means algorithm.

### 4.3. Speedup Analysis

This section analyzes the performance of the parallel *K*-means algorithm in terms of speed ratio. Speed ratio is one of the important criteria to measure the performance of parallel computing. It describes the overall performance improvement achieved by shortening the running time of algorithm parallelization in clustered environment. The calculation equation of the speed ratio is given in the following equation:

(4) $$\begin{array}{c} E=\frac{T_{s}}{T_{r}}, \end{array}$$

where *T*_*s*_ represents the time it takes for the algorithm to run under a single node, and *T*_*r*_ represents the time it takes for the algorithm to run in a distributed cluster environment composed of *r* nodes with exactly the same performance. As shown in Figure 5, the speed ratio of parallel *K*-means algorithm of all 3 datasets is the same. We can observe from Figure 5 that speed increases with increasing the number of nodes for all 3 datasets.

## 5. Conclusion

This study proposes to use the Spark framework based on memory computing to enhance the effect of basketball data analysis. The proposed framework has better execution efficiency by introducing the cuckoo search algorithm in the emerging swarm intelligence optimization method. The findings from experiments show that the method in this study is faster and more useful in practical applications than other methods. The shooting training effect in the active area has the most measurable impact and has a good influence on the training effect. In fact, given that big data will be playing an increasingly significant role in sports in the next several years, legal protection problems of this type of particular information will only become more important in the future.

## Figures and Tables

**Figure 1:** Spark's overall architecture.

**Figure 2:** The core composition of Spark.

**Figure 3:** Schematic diagram of *K*-means clustering algorithm.

**Figure 4:** Scalability analysis of the proposed model.

**Figure 5:** Comparison results of parallel *K*-means algorithm speedup.

**Table 1:** Apache Spark configuration detail of cluster.

Specification	Processor	3.20 GHz × 10
	Connectivity	100 Mbps Ethernet LAN
	Hard disk	1 TB
	Memory	250 GB
	CPU	Intel Core Tm

Software	Operating system	Ubuntu 18 LTS
	Hadoop	2.7.3
	OS type	64 bit
	Spark	2.3.4
	Java development kit	16

**Table 2:** Cluster execution time of each algorithm (sec).

Test datasets	DATA1		DATA2		DATA3	
	Shortest	Longest	Shortest	Longest	Shortest	Longest
Serial *K*-means clustering	12.36	28.65	32.89	50.12	1025.66	1574.23
Parallel *K*-means clustering	40.65	54.23	99.36	124.32	589.36	851.36

## Data Availability

The data used to support the findings of this study are included within the article.
